This article has been retracted.

# Meta-Analysis of Different Acupuncture Points in the Treatment of Ankylosing Spondylitis with Supervised Moxibustion

**DOI:** 10.1155/2022/4688689

**Published:** 2022-10-11

**Authors:** Jie Cheng, Xinyi Wang, Leisheng Wang, Yufei Zhang, Yu Gu, Dan Mao, Xingyu Zhou, Xiaolong Wang, Yuansheng Tian

**Affiliations:** ^1^College of Henan Traditional Chinese Medicine, Zhengzhou 450000, Henan, China; ^2^The Affiliated Hospital of Henan Academy of Traditional Chinese Medicine, Zhengzhou 450000, Henan, China

## Abstract

**Objective:**

To investigate the clinical efficacy of different acupuncture points in the treatment of ankylosing spondylitis with supervised moxibustion.

**Methods:**

Retrospective analysis of 61 AS patients (diagnosed as ankylosing spondylitis of kidney-yang deficiency type by Chinese medicine) admitted to our hospital from January 2020 to February 2021, randomly divided into 30 cases in the experimental group (Du moxibustion + basic western medicine treatment) and 31 cases in the control group (basic western medicine treatment alone). The changes in quantitative scores of the main symptoms and major signs (thoracic mobility, occipital-wall distance, finger-ground distance, and laboratory index (ESR)) were analyzed before and after treatment.

**Results:**

Of the 30 cases in the experimental group, 2 were clinically cured, 3 were apparently effective, 21 were effective, and 4 were ineffective, with an overall effective rate of 86.7%; of the 31 cases in the control group, 1 was clinically cured, 1 was apparently effective, 1 was effective. 24 were effective, and 5 were ineffective, with an overall effective rate of 83.9%. Comparing the efficacy by *t*-test, *P* < 0.05, indicating that the effect of Du moxibustion + Western medicine treatment was better.

**Conclusion:**

The treatment of ankylosing spondylitis with kidney-yang deficiency by moxibustion + western medicine can improve the efficacy, alleviate the inflammatory response and improve the patient's symptoms and signs, and immune indexes.

## 1. Introduction

Ankylosing spondylitis (AS) is a chronic progressive immune inflammatory disease with undetermined pathogenesis. It mainly affects the medial and peripheral joints of the human body, manifesting mainly as synovial inflammatory lesions of the joints, followed by deformation and destruction of the cartilage, and eventually developing into bony ankylosis and vertebral joint-like changes, as well as involving the eyes, heart, lungs, and kidneys. It may also involve the eyes, heart, lungs, kidneys, and other organs. The early manifestations are mainly pain in the sacroiliac joints, and the onset of the disease is relatively insidious, but because of the late start of rheumatological research in China and the lack of attention to rheumatic diseases, the diagnosis is often unknown or late. Epidemiological surveys have shown that there are significant ethnic and regional differences in the disease, with a prevalence of 0.3% in China and a predominantly adolescent population with a male to female ratio of 2 : 1. In China, 60% of patients with ankylosing spondylitis have hip involvement, and 15–20% have bony ankylosis of the hip joint, or even lifelong disability [1, 2], which causes great pain to the patient's work and life, and is a serious burden to the family and society, so research into this disease is of great significance.

Ankylosing spondylitis is not known as a disease in traditional Chinese medicine, but there are many records relating to it. It can also be classified as “paralysis” or “lumbago.” From the perspective of Chinese medicine, the causes are internal and external. The internal cause is mainly a deficiency in the kidney [2], which is responsible for the production of bone and marrow. The kidney is the innate essence of the human body, and all physiological functions of the human body depend on the fullness of kidney qi. The Kidney is also the innate essence of the human body and all physiological functions of the body depend on the fullness of Kidney Qi. The Governor's Vessel oversees the Yang Qi of the body and is the sea of Yang Qi. The main external causes of the disease are closely related to “cold and dampness.” In Su Wen's Theory of Paralysis, the three gases of wind, cold, and damp come together and become paralysis.

The insidious onset of ankylosing spondylitis and the atypical early symptoms make it easy to confuse the disease with other diseases, presenting a significant obstacle to early diagnosis and treatment. The treatment of AS has not yet been found to be curative, and the goal of treatment remains to control the disease, reduce pain and mobility restrictions to the greatest extent possible, prevent bone damage to the joints and restore mobility to the spinal joints. The first-line drugs used in Western medicine to treat AS are still mainly NSAIDs, antirheumatic drugs, anti-TNF antagonists, and glucocorticoids, with the rest being thalidomide and leflunomide, which are not as effective as the first-line drugs, while hip replacement surgery is less acceptable to patients because of the greater risk of postoperative heterotopic ossification. Moreover, the long-term application of NSAIDs is extremely damaging to patients' gastrointestinal tract and liver and kidney functions. The treatment of AS in Chinese medicine is based on the principle of evidence-based treatment and is classified according to the causes and symptoms of the disease, which are mostly classified into cold-damp paralysis and obstruction, damp-heat paralysis, stasis-blood paralysis, and obstruction. The internal treatment method is based on traditional Chinese medicine soup or Chinese medicine pills processed according to the Chinese medicine formula, which are effective in reducing joint pain and improving joint function in AS. The external treatment of ankylosing spondylitis is based on a variety of methods, such as acupuncture, moxibustion, acupuncture, Gua Sha, compressing, fumigation, and Tui Na, which are fast acting, effective, and reduce the side effects of oral medication.

The insidious onset of ankylosing spondylitis and the atypical early symptoms make it easy to confuse the disease with other diseases, presenting a significant obstacle to early diagnosis and treatment. The treatment of AS has not yet been found to be curative, and the goal of treatment remains to control the disease, reduce pain and mobility restrictions to the greatest extent possible, prevent bone damage to the joints and restore mobility to the spinal joints. The first-line drugs for the treatment of AS in Western medicine are still mainly NSAIDs, antirheumatic drugs, anti-TNF antagonists, and glucocorticoids, and the rest are thalidomide and leflunomide, which are not ideal for first-line drug effects, while hip arthroplasty is less acceptable to patients due to the greater risk of postoperative heterotopic ossification [3, 4]. Moreover, the long-term application of NSAIDs is extremely damaging to patients' gastrointestinal tract and liver and kidney functions. The treatment of AS in TCM is based on the principle of evidence-based treatment, is classified according to the etiology and symptoms of the disease, and is mostly divided into evidence types such as cold-damp paralysis and obstruction, damp-heat paralysis, stasis-blood paralysis, and obstruction. The internal treatment method is based on traditional Chinese medicine soup or Chinese medicine pills processed according to the Chinese medicine formula, which are effective in reducing joint pain and improving joint function in AS. There are many external treatments for ankylosing spondylitis, such as acupuncture, moxibustion, acupuncture, Gua Sha, compressing, fumigation, and Tui Na, which are fast acting and effective and reduce the side effects of oral medication.

Chinese medicine treatment is mainly based on the identification and treatment of positive deficiency, evil actuality, and mixed deficiency and actuality, using Chinese medicine's internal and external treatment methods, but the efficacy is limited [5, 6]. If the kidney yang is deficient, the fire of the vital gate is insufficient, the source of the Governor's Vessel is depleted, and the warming power is weak; if the Governor's Vessel is blocked, the circulation of Qi and blood is poor, and the ability to resist external evil is reduced. In recent years, studies have found that the treatment of ankylosing spondylitis with moxibustion is effective, improving clinical symptoms and relieving fatigue [7, 8]. However, there are shortcomings in the treatment of ankylosing spondylitis, such as uneven heat distribution, low drug utilization rate, and easy-to-burn patients. The moxibustion box is a kind of warm moxibustion apparatus that can effectively use the smoke and heat produced by burning moxa, and by fumigating or warming certain parts of the body surface, it can adjust the function of meridians and internal organs, thus playing a role in disease prevention and treatment. In this study, moxibustion was applied to patients with ankylosing spondylitis with a deficiency of kidney yang in order to provide a basis and new ideas for the adjunctive treatment of ankylosing spondylitis.

## 2. Materials and Methods

### 2.1. Source of Cases

Patients with AS who were admitted to our hospital from January 2020 to February 2021 (with a TCM diagnosis of renal yang deficiency building) were selected. A total of 63 cases met inclusion criteria, 2 cases dropped out during the treatment period, and 61 cases completed the course of treatment. The gender ratio was 43 males and 18 females; age ranged from 19 to 65 years old, with an average age of 40 years old; income cases The course of disease ranges from 1 to 10 years, with an average of 5 years. According to the random number table, patients were randomly divided into two groups: experimental and control.

### 2.2. Diagnostic Criteria of Western Medicine

Western medicine diagnosis is based on the AS criteria in China's 2002 Guidelines for Clinical Studies of New Western Medicines. The main symptoms are lumbosacral pain, back pain, restricted spinal movement, joint swelling not exceeding the surrounding bony signs, and morning stiffness; the main signs are tenderness at the attachment point, Schober test (+), positive occipital wall, finger test, positive, or normal thoracic range of motion; X-ray film shows mild Inflammatory infiltrate with indistinct contours, dense shadows around the joint, and a slightly smaller interarticular space.

### 2.3. Chinese Medicine Syndrome Differentiation Criteria

The TCM typology of ankylosing spondylitis is based on the Guidelines for Clinical Research on New Chinese Medicines. Kidney-yang deficiency syndrome's primary symptoms are as follows: back pain, back pain, restricted lumbar spine movement, morning stiffness, local cold pain, aversion to cold and warmth, lack of warmth in the hands and feet, heel pain, and soreness and weakness of the waist and knees. Secondary symptoms are as follows: lack of energy, pale complexion, soreness and weakness of the waist and knees, impotence, and excessive nocturia. Tongue and pulse: pale tongue with white fur and deep and thin pulse.

### 2.4. Quantitative Scoring Criteria for Major Symptoms

The quantitative scoring standard of main symptoms in this experiment is based on my country's “Trial Implementation of Principles for Guiding Clinical Research on New Chinese Medicines” and is prepared according to specific clinical manifestations of clinically collected patients.

### 2.5. Inclusion Criteria

The inclusion criteria were set as follows:

1. Previously diagnosed with ankylosing spondylitis, with a history of more than 1 year and no more than 10 years
2. Conform to TCM syndrome differentiation of ankylosing spondylitis with kidney-yang deficiency syndrome
3. Aged between 19 and 65 years old
4. After informing the patient of a specific treatment plan, he is still willing to accept 2 courses of treatment, and cooperates with a relevant examination, as evidenced by signing “informed consent”

### 2.6. Exclusion Criteria

The exclusion criteria were set as follows:

1. Ankylosing spondylitis is not clearly diagnosed; those who do not meet TCM classification criteria for kidney-yang deficiency
2. Age < 19 or > 65 years old; female patients during menstruation, pregnancy or lactation
3. Patients with other joint diseases coexisting with negative rheumatoid factor accompanied by more serious chronic primary underlying diseases such as hypertension, disease, coronary heart disease, diabetes, blood with coagulation, hematopoietic, and other disorders; patients with systemic diseases; patients with mental or unconscious problems
4. Patients with severe joint deformities or even disabilities;
5. Those who refuse to cooperate with researchers, or have incomplete clinical data, which may affect the statistics of research results

### 2.7. Rejection Criteria

The rejection criteria were set as follows:

1. After inclusion, it was found that patient concealed their condition but did not actually meet the inclusion criteria to be selected
2. Those who have poor compliance, do not follow doctor's orders for a course of treatment, and refuse to cooperate with treatment and inspection
3. Other conditions that may affect the results of this treatment occur during the study period

### 2.8. Falling off Standard

The following cases are regarded as dropout cases: those who drop out of an incomplete course of treatment due to the patient's own reasons (work or personal reasons); those who drop out of an incomplete course of treatment due to serious discomfort with Du moxibustion during the course of treatment.

### 2.9. Research Content

Based on the principle of randomized control, clinical treatment of Du moxibustion in the treatment of ankylosing spondylitis (kidney-yang deficiency type) was observed. A total of 63 cases meeting inclusion criteria were collected in Min 2.2 grouping, and they were randomly divided into an order of hospitalization time and random number (table. 2) groups: experimental (the Governor's moxibustion + western medicine basic treatment), control (simple western medicine basic treatment). During the course of treatment, 1 case dropped out in experimental and control, respectively, so a total of 30 cases were completed in experimental and 31 cases in control.

### 2.10. Treatment Methods

Experimental: Governor's moxibustion + basic western medicine treatment.

*Specific Operations*. Acupuncture: the patient is placed in a prone position, and Hua Lun Jiaji acupoint is selected, that is, under a spinous process of 1st thoracic vertebra to 5th lumbar vertebra, 0.5 cun on the left and right sides, 17 acupoints on each side, a total of 34 acupoints. Disposable sterile governor moxibustion needles were punctured obliquely at 45° in direction of the spine, needles were inserted 15 mm, and needles were retained for 30 min. For 6 consecutive days, once a day, and on the 7th day, Du moxibustion was performed. On the 7th day, supervisor moxibustion: take an appropriate amount of small turmeric, wash it, crush it with a juicer, then take out the crushed ginger paste, wrap it in gauze, squeeze out a little ginger juice, and instruct the patient to lie on the bed, fully expose spine, use iodine disinfect local skin of T, ∼Ls, lay a layer of gauze, and then lay ginger mud, about 5 cm wide and 1.5 cm thick, and place moxa columns (diameter 1.5 cm) on it, with an interval of about 2 cm between each column. After burning, the next column was replaced, and a total of 3 columns were continuously applied for moxibustion, as shown in Figure 1. For 1 month after moxibustion, do not take cold water baths and fast food. Acupuncture treatment was continued after Governor's moxibustion, and this cycle of treatment, every 2 weeks was a course of treatment, a total of 4 courses of treatment, and a total of 2 months of treatment.

Western medicine basic treatment: oral celecoxib capsules (produced by China Pfizer Pharmaceutical Co., Ltd.), 1 tablet (0.2 g) each time, once a day. 1 week is a course of treatment, and a total of 2 courses of treatment are taken. Control: only received basic western medicine treatment. 1 week is a course of treatment, and a total of 2 courses of treatment are taken. Care measures: advise patients to eat a diet high in nutrients and vitamins, light and easy to digest; advise patients with noncardiopulmonary insufficiency to take appropriate spinal and joint function-based exercises; and advise patients to sleep on a hard bed.

### 2.11. General Observation Indicators

The evaluation of the efficacy of ankylosing spondylitis was carried out according to the assessment of ankylosing spondylitis (ASAS) [9], and the thoracic mobility, finger-to-floor distance, occipital-wall distance, and Schober test were evaluated before and after treatment in both groups.

Laboratory parameters: early morning fasting venous blood was collected from both groups before and after treatment by the same nursing staff and sent to the hospital's laboratory department for testing. The interleukin-17 (IL-17) and interleukin-1*β* (IL-1) samples were sent to the laboratory department of the hospital. The erythrocyte sedimentation rate (ESR) of all samples was measured by a fully automatic dynamic sedimentation analyzer (purchased from Shenzhen Yafei Long Biotechnology Co. protein (CRP) levels were measured with a fully automated hematology analyzer (purchased from Shenzhen Meizu Biomedical Electronics Co.

### 2.12. Main Symptoms

Based on my country's 2002 “Principles for Guiding Clinical Research on New Chinese Medicines,” based on self-made scoring standards based on the main symptoms of clinical patients, patients' lumbosacral, back pain, spinal activity, and other symptoms were evaluated. Finally, the total score was used to compare the improvement of the main symptoms.

### 2.13. Main Signs

The thoracic activity, occipital-wall distance, and finger-ground distance (cm) of patients were measured and recorded for comparison.

### 2.14. Laboratory Indicators

After admission, patients underwent serum ESR detection in our hospital, and changes in erythrocyte sedimentation rate (mm/h) were compared.

### 2.15. Criteria for Determining Clinical Efficacy

After the clinical rash, symptoms of lumbosacral and back pain disappeared or basically disappeared, and the range of motion of spinal joints was basically normal. The activity of the chest seat increased by > 2.5 cm, the pillow-to-wall distance decreased by > 10 cm, and the finger-to-ground distance decreased by >10 cm. ESR reduction > 10 mm/h. The symptoms of lumbosacral and back pain were relieved, and the range of motion of spinal joints was improved. Thoracic range of motion > 1 cm and < 2.5 cm, pillow-to-wall distance decreased by > 5 cm and < 10 cm, and finger-to-ground distance decreased by >5 cm and <10 cm. ESR > 5 mm/ho improved, lumbosacral and back pain symptoms were relieved, spinal joint mobility improved, chest gallery mobility slightly improved, the occipital-wall distance decreased by > 10 cm, and finger-ground distance by > 10 cm. The ESR results were slightly improved. There was no change in ineffective symptoms compared with those before treatment. Effective rate = cure + marked effect + improvement.

### 2.16. Criteria for Judging Efficacy of Syndromes

The clinical symptoms related to TCM basically disappeared, and the quantitative score of symptoms decreased by >90%. The symptoms related to TCM with marked effect were improved, and the symptom quantitative score decreased by >70%. Effective TCM-related symptoms were improved, and the symptom quantitative score decreased by > 30%.

### 2.17. Quality Control

1. Design the experiment rigorously and reasonably, and comprehensively collect theoretical data supporting the experiment
2. A clinician who did not participate in the treatment operation of this experiment measured and recorded various clinical indicators, and evaluated TCM symptoms strictly according to self-made scoring standards
3. Provide professional training to experimental operators, formulate clear operating specifications and experimental procedures, and conduct experiments in accordance with standardized operations during treatment;
4. The final data are statistically analyzed with professional software
5. The experimental operation is always carried out by one person to prevent experimental results from being affected by deviation of acupoint selection method or irregular operation

### 2.18. Statistical Methods

SPSS 21.0 statistical software was used for statistical analysis and processing of the data. The mean ± standard deviation ($\bar{x}\pm s$) was used for measurement data. *α* = 0.05, *P* < 0.05 is considered a statistically significant difference.

## 3. Results

Among 63 AS patients, there were 45 males and 18 females; random serial numbers were obtained from a random number table, and cases were randomly divided into two groups by the remainder method. There were 30 cases and 31 cases in control. The age, gender, and duration of disease were compared. See Table 1.

A nonparametric test was used for curative effect, indicating that the total effective rate of experimental was better. See Table 2.

The *t* test was used to analyze quantitative scores of the main symptoms of patients. The curative effect of the experiment was better; a comparison of each was performed by *t*-test, and results showed that scores after treatment were lower than those before treatment. See Table 3.

By comparing changes in a thoracic range of motion, occipital-wall distance, and finger-to-ground distance of patients, results were statistically analyzed, and *t*-test was used to compare. The curative effect of the experiment was better; see Tables 4–6.

The *t*-test was used to analyze ESR changes. The results showed that there was a difference in ESR after treatment (*F* = 9.611, *P* < 0.05), and the curative effect of the experiment was better. See Table 7.

## 4. Discussion

The results of this study showed that the moxibustion intervention in the moxibustion box of the Governor's Vessel was effective in improving the TCM symptoms and signs of patients with ankylosing spondylitis. The basic pathogenesis of ankylosing spondylitis is that the patient has congenital deficiencies and deficiencies in the Governor's Vessel and kidney channels. In modern Chinese medicine, clinical trials suggest that the kidneys and the Governor's Vessel are the basis of ankylosing spondylitis, with the Governor's Vessel running through the entire spine and connecting to the kidneys, and the Governor's Vessel unifying the Yang of the body. If the disease is not treated for a long period of time, it will become a condition where “the jib takes the place of the heel and the spine takes the place of the head” (Su Wen-Theory of Paralysis). “Kidney deficiency and stagnation of the Governor's Vessel are the main causes of this condition. A deficiency of kidney yang leads to insufficient fire in the vital gate, depletion of the source of the Governor's Vessel, and weakness in warming power. Moxibustion interventions in the moxibustion box of the Governor's Vessel can tonify the kidneys and open up the channels and meridians, stimulating and strengthening the warmth of Yang, which in turn promotes the flow of Qi and blood, ultimately achieving the purpose of unblocking the Qi flow, harmonizing Qi and blood, and restoring physiological functions [10, 11]. By warming the yang of the body, the warming effect of kidney qi is used to nourish the kidney essence, which in turn enriches the bone marrow, thereby improving the local and general symptoms of ankylosing spondylitis, and its clinical effects have been confirmed.

The results of this study showed that after treatment, the thoracic mobility and Schober's test scores were higher in the observation group than in the control group, and the finger-ground and occipital-wall distances were lower than in the control group (*P* < 0.05). Sacroiliitis is a hallmark of ankylosing spondylitis, which can be characterized by bone and articular cartilage defects in the early stages and spinal deformities and ankylosis in the later stages, with severe limitations in functional activity. The moxibustion box is a warm moxibustion apparatus, when moxibustion is ignited in the box, it allows the moxa to burn fully to produce smoke and heat, which can burn or warm the patient's body surface, thus playing a role in regulating the function of the meridians and organs and playing a curative role. A study [12] used supervised moxibustion combined with oral salazapyridine tablets to treat ankylosing spondylitis and showed that compared with acupuncture combined with oral salazapyridine tablets, supervised moxibustion combined with oral salazapyridine tablets treatment could significantly improve the symptoms and signs of patients with ankylosing spondylitis with deficiency of kidney yang. Some studies have shown that ginger-garlic supervision and moxibustion can significantly improve the signs and bone metabolic indexes of patients with ankylosing spondylitis with a deficiency of kidney yang [13, 14]. The results of this study showed that the signs improved in both groups after treatment, but the observation group was better than the control group. It may be that the warm stimulation of the moxibustion box moxibustion therapy of the Governor's vein can better stimulate the body's ability to resist disease.

Moxibustion can remove blood stasis and activate blood, improve blood rheology, correct free radical metabolism disorders, and can inhibit the release of inflammatory cytokines, and enhance the body's immune function [15, 16]. The results of this study suggest that the levels of IL-1, IL-17, CRP, and ESR in the observation group were lower than those in the control group after treatment (*P* < 0.05). IL-1, IL-17, CRP, and ESR are common indicators of the inflammatory response. IL-17 can further induce pro-inflammatory cytokine expression, causing and exacerbating inflammatory cell infiltration and tissue damage [17, 18]. Studies have shown that moxibustion can effectively reduce inflammatory indicators such as CRP and ESR, which is consistent with the results of this study [19, 20]. The moxibustion box can regulate the body's immune response and endocrine, effectively controlling the inflammatory response and improving the therapeutic effect of ankylosing spondylitis [21].

The combination of moxibustion and moxibustion box moxibustion can stimulate and strengthen the Yang energy to warm the body and then promote the flow of Qi and blood, ultimately achieving the purpose of clearing the Qi flow, harmonizing Qi and blood, and restoring physiological functions, thus effectively improving the therapeutic effect, relieving the inflammatory response and improving clinical symptoms. There are still shortcomings in this study, such as the small sample size, the short duration of the study design, and the single type of evidence. There is a need to further expand the sample size and conduct in-depth studies on different types of patients.

## Figures and Tables

**Figure 1:** Schematic diagram of supervisor moxibustion method.

**Table 1:** Comparison of general conditions of patients.

Grouping	Number of cases	Age ($\bar{x}\pm s$, years)	Gender		The course of disease ($\bar{X}\pm S$, year)
			Male	Female	
Treatment	30	39.93 ± 10.52	20	10	4.77 ± 3.06
Control	31	40.06 ± 10.64	23	8	6.16 ± 2.88

**Table 2:** Comparison of curative effects of patients (cases).

Group	*n*	Recovery	Remarkable effect	Valid	Invalid	Efficiency (%)
Treatment	30	2	3	21	4	86.7
Control	31	1	1	24	5	83.9

**Table 3:** Comparison of quantitative scores of main symptoms of patients ($\bar{x}\pm s$).

Group	*n*	Before treatment	After treatment
Treatment	30	26.95 ± 3.90	11.2 ± 4.21
Control	31	25.05 ± 3.37	13.62 ± 3.68
*F*-value		1.085	2.593
*P*-value		0.304	0.02

**Table 4:** Comparison of thoracic range of motion ($\bar{x}\pm s$).

Group	*N*	Before treatment	After treatment
Treatment	30	2.48 ± 0.86	4.18 ± 1.51
Control	31	1.95 ± 0.79	2.5 ± 0.96
*F*-value		1.162	5.821
*P*-value		0.285	0.019

**Table 5:** Comparison of occipital-wall distance ($\bar{x}\pm s$).

Group	*N*	Before treatment	After treatment
Treatment	30	6.886.27	3.09 ± 4.67
Control	31	5.27 ± 4.13	4.02 ± 3.94
*F* value		1.483	1.982
*P* value		0.226	0.049

**Table 6:** Comparison of the finger-ground distance ($\bar{x}\pm s$).

Group	*N*	Before treatment	After treatment
Treatment	30	23.44 ± 10.86	15.95 ± 8.44
Control	31	24.92 ± 14.02	19.18 ± 12.35
*F* value		1.482	5.765
*P* value		0.227	0.022

**Table 7:** Comparison of ESR ($\bar{x}\pm s$).

Group	*n*	Before treatment	After treatment
Treatment	30	14.05 ± 10.53	8.79 ± 7.68
Control	31	20.86 ± 20.32	12.86 ± 16.05
*F* value		0.754	9.613
*P* value		0.454	0.005

## Data Availability

The experimental data used to support the findings of this study are available from the corresponding author upon request.
